The article "Nutrient intake, alcohol consumption, emotional eating and anxiety in women nursing students" was published in 2023. Journal: Heliyon.

# Nutrient intake, alcohol consumption, emotional eating and anxiety in women nursing students

**DOI:** 10.1016/j.heliyon.2023.e22903

**Published:** 2023-11-30

**Authors:** María Teresa Iglesias López, Carlos Alberto Marchena-Giráldez, Elena Bernabéu-Brotons

**Affiliations:** a Facultad de Ciencias de la Salud. Universidad Francisco de Vitoria, Spain; b Facultad de Educación y Psicología. Universidad Francisco de Vitoria, Spain

**Keywords:** Nursing students, Alcohol consumption, Habits, Anxiety, Nutrients, Emotional eating

## Abstract

**Objective:**

The aim of the study was to analyze dietary habits, alcohol habits, emotional eating and anxiety in a sample of Spanish nursing students. These students appear to be essential to the field of public health and to teaching their future patients about their own good practices.

**Methods:**

A cross-sectional investigation was conducted. Participants completed the Emotional Eater Questionnaire, the Alcohol Use Disorder Identification Test (AUDIT) test to evaluate alcohol intake, the State-Trait anxiety Inventory (STAI) test to measure levels of anxiety as a state and anxiety as a trait, and self-reported sociodemographic data. Following classroom instruction, three-day food records were used to gauge food intake.

**Results:**

The calorie intake for the macronutrients Ca, Mg, K, and Fe were below the Recommended Dietary Intakes (DRI) and imbalanced. The percentage E of proteins was 132.7 % more than recommended, while the percentage of carbohydrates is below the recommended level. Dietary energy consumption barely equaled 78 % of the total energy consumed by this sex and age group. With respect to emotional eating, nursing women students were low emotional eater (44 %) > emotional eater (30 %) > non-emotional eater (22.7 %). The students' emotional eating is substantially connected with fast food and sweets, or less healthy food intake behaviors. According to the Alcohol Use Disorder Identification Test (AUDIT), 82.7 % of female students used alcohol on a regular basis in a low-risk manner.

**Conclusion:**

The findings demonstrated a link between anxiety and dietary fat intake. Trait anxiety was negatively connected with emotional eating (EE), whereas state anxiety was positively correlated with meat consumption. It is crucial to consider these findings when creating prevention/intervention plans and profiles of harmful eating behaviors.

## 1 Introduction

• Nursing students continuously learn about health promotion in the nursing curriculum and as future healthcare professionals. These students are crucial to the field of public health. As Hwang noted, it's crucial to educate nursing students about their own health since they understand the value of adopting health-promoting habits while receiving their education and because they exhibit the same bad habits as other students [1]. Identification and modification of positive and negative health habits contributing to subjective and physical well-being could help prevent the onset of lifestyle-related illnesses and improve quality of life [2]. Due to their skills in providing patients with the best care possible, nursing students should recommend holistic health practices to patients to improve their psychological well-being and quality of life. The promotion of positive shifts in nurses' attitudes, beliefs, and levels of confidence towards bad eating habits can be achieved by educating interventions [3]. Eating behaviors, different between individuals, are the most influential factor in the development of chronic pathologies and diet is one of the most significant healthiest defining it. In this way, high adherence to a healthy diet has the future potential to prevent disease and most studied healthy dietary pattern was the Mediterranean [3].

The article "Nutrient intake, alcohol consumption, emotional eating and anxiety in women nursing students" was published in 2023. Journal: Heliyon.

A healthy diet plays a crucial role in preventing chronic diseases such as obesity, type 2 diabetes, cardiovascular diseases, and certain types of cancer [4].. The current dietary patterns from the university students are moving away from the traditional Mediterranean diet and comprise a higher intake of animal instead of vegetal products such as legumes, nuts, fruits, and vegetables. Healthy eating and meal preparation are often sacrificed and replaced by convenience and junk foods and excessive alcohol consumption during this time of life and may influence other habits like eating habit [5,6].

The scientific community has demonstrated the significance of a healthy diet based on Mediterranean dietary patterns for the psychological system, due its potential means of decreasing the risk of anxiety and depression, especially in young adults [7]. This pattern is linked to a culinary culture and traditions [8]Energy intake as well macro and micronutrients intake (carbohydrate, protein, calcium, iron, zinc, vitamin A, thiamin, and riboflavin) are associated with cognitive performance in young women [9,10]. Mediterranean diet pattern is characterized by high intake of vegetables, fruits, nuts, cereals, legumes and olive oil as the principal source of fat, moderate to-high-intake of fish, moderate consumption of dairy products and wine (during meals) and low consumption of meat and poultry [11], and contains low total fat, low saturated fat, and high monounsaturated fatty acid: saturated fatty acid (represented by the omega-6 and omega-3).

Adherence to Mediterranean diet, may have a possible positive effect on wellbeing, cognition sleep pattern protecting against psychological diseases, which is important in university students [[12], [13], [14], [15], [16], [17], [18]].

The article "Nutrient intake, alcohol consumption, emotional eating and anxiety in women nursing students" was published in 2023. Journal: Heliyon.

Is has been observed that a diet rich in omega-3 and omega-6 is effective in reducing anxiety and prevents anxiety symptoms [[19], [20], [21], [22]] Similar results presented that fruit and vegetable consumption has positive effects on mood, reducing the level of psychological distress [23]. It also has been found that people from the general population with mood and anxiety problems showed less anxiety and perceived stress after a supplementation with multivitamin/multimineral formulas and B complex vitamins [24] [27 or increasing their intake of vitamin D [25]. In a study carried out with nurses, higher levels of stress were associated with a higher energy intake and a higher percentage of fat and saturated fat [26].

The degree of adherence of Spanish university students to MD has been the subject of several research [[27], [28], [29]] which have used the Mediterranean Diet Quality Index (KIDMED) questionnaire [30]. Spanish university population with lower degree of adherence is related to problems of mental health and higher levels of negative emotions, such as stress, anxiety, and, consequently, lower self-esteem [31]. By contrast, greater adherence to MD combined with greater socialization reduces the risk of depression by some 50 % [24,32].

Many students leaving their home to obtain a Degree were under academic pressure and worry about academic performance and this can be a cause of depression, anxiety and stress [33,34]. [35]. during university studies. The increased of anxiety is associated with poor sleep. , It has been proven that stress reduction improves both anxiety and sleep [36,37]. The absence of effective strategies to deal with negative emotions may result in the adoption of inappropriate or harmful coping mechanisms such as alcohol consumption as a coping strategy especially for anxiety [38] or unhealthy eating patterns as emotional eating [39]. , s an automatic response to negative emotions [40,41].

Students’ academic performance is also affected by a multitude of factors as the consumption of fish, milk, fruits, and vegetables. Burows et al. (2017) reported that dietary patterns seem to be more strongly associated with cognition than individual foods, probably due to the synergistic effects of each food component [42]. High or more frequently low food intake may be more likely during and directly after a drinking occasion, a consequence related with this alcohol drinking to avoid weight gain, because alcohol contains empty calories and does not stimulate satiety [43,44]..

The article "Nutrient intake, alcohol consumption, emotional eating and anxiety in women nursing students" was published in 2023. Journal: Heliyon.

There are some studies that emphasized the relationship between short sleep duration and poor dietary intake or influences dietary composition: fewer servings of fruits vegetables, whole grains and beans and overall poorer dietary quality [45]. Also, it has been observed that relative to normal sleepers (7–8 h), short sleepers (5–6 h) reported higher intakes of absolute protein, carbohydrate, and total fat but a lower intake of dietary fiber, whereas very short sleepers (<5 h) reported lower intakes of protein, carbohydrates, dietary fiber, and total fats [46]. In a study of adolescents across several European countries, those who slept <8 h were more sedentary and demonstrated a decrease of healthy foods intake [47,48]. It has been observed that shorter sleep durations are associated with unhealthier dietary habits or skipping breakfast [[49], [50], [51], [48]]. Poor sleep quality and quantity has been associated with impaired health and academic performance. Diet quality has been studied with respect sleep [52]. The number of studies investigating the role of [51]individual dietary factors and overall dietary patterns toward depressive, anxiety, and sleep disorders provide an interesting body of evidence and the dietary intake of specific nutrients such as n-3 polyunsaturated fatty acids, B vitamins, zinc, and magnesium have been implicated in brain function. B-group vitamins may modulate cognitive performance and improve cerebral and cognitive [32,53,54].

1. To analyze dietary habits, alcohol habits, emotional eating, and anxiety in a women Spanish university nursing students sample
2. To determine if anxiety and emotional eating were related to dietary habits.

## 2 Material and methods

1. Study, Participants and Procedure

This cross-sectional study was performed during October–December 2019 with a sample of 250 women students from Nursing Degree of first and second year of their studies. The Nutrition Professor provided information to the students about the study, after those 200 students agree to participate in this study and the final sample was 150 women, men were excluded because there were scarce represented. Before beginning the study, written informed consent was sought from those who intended to participate. Convenience non-aleatory sample was used. The study protocol and design were approved by the Ethics Committee of the University Francisco de Vitoria (17/2019), and it fully complied with the Helsinki Declaration. The evaluation protocols were provided physically, and the data was uploaded onto a database for analysis. The data were collected during scholar hours with any incidents and analyzed anonymously. The academic aspect was calculated by average mark for each student during their academic career, for this each student was asked for the marks obtained during their Nursing study.

The article "Nutrient intake, alcohol consumption, emotional eating and anxiety in women nursing students" was published in 2023. Journal: Heliyon.

As an inclusion criterion, it was first-year or second-year students of Nursing Bachelor. Exclusion criteria were based on age (18 students >25 years), missing data (14 students), as well as low energy intake (either too low or too high) which was determined by Goldberg cut-off points. Finally, a total of 150 subjects (Fig. 1) completed the study with a mean age of 20 ± 2.0 years.

2. Questionnaires

**Fig. 1:** Flow-chart of the study.

Participants completed self-reported sociodemographic information on their age, course, nationality, height, weight. The methodology employed in the study was previously explained [55,56].

a) Dietary assessment and Adherence to Mediterranean Diet

Food intake was assessed using three-day food records (two weekdays and one weekend day), after receiving training in class time. The dietary intake of a selection of nutrients: energy, macro and some micronutrients, was compared with age and sex-specific requirements of these nutrients according to the dietary recommended index (DRI) for Spanish population [57]. The number of nutrients with inadequate intake was determined for each participant. Energy and nutrient intakes were determined using Spanish DIAL® software. Food frequency consumption was evaluated according to a six-point scale: (1) daily, (2) 4 to 6 times a week, (3) 2 to 3 times a week, (4) once a week, (5) frequently, (6) never”. These frequencies were converted into metric data (times per day), ranging from: 2, 1, 0.5, 0.14, 0.06 and 0 times/day of different food groups, including meat, fish, legumes, fast food, snacks, fried foods, alcohol, soft drinks, as well as daily consumption frequency of milk products [57].

b) Alcohol consumption

To assess alcohol consumption and behavior, the three-item screening tool, Alcohol Use Disorders Identification Test, or AUDIT-C, was used. The AUDIT-C is a short version of the 10-question AUDIT (screening tool developed by the World Health Organization to assess alcohol consumption, drinking behaviors and alcohol-related problems [58,59]. The AUDIT test was used to determine the alcohol consumption habits of the participants. Audit test Cronbach alpha was 0.93 (95 % confidence interval [CI], 0.921–0.941). The test consists of 10 items, 8 of which are on a Likert scale of 5 categories 24 ordered from 0 (never/1 or 2 units) to 4 (daily/10 or more units). The two remaining items also use a Likert scale but with 3 categories ordered from 0 to 2. The response from participants allows them to be classified into three levels: without risk of dependence, at risk consumption and probable alcohol dependence syndrome (ADS). AUDIT-C uses the first three questions, is sensitive and specific properly to be a valid tool for identifying high-risk consumption. The recent validation of both the AUDIT and the AUDIT-Con Spanish university population carried out by García et al. [60] found the internal consistency of the AUDIT test to be α = 0.75, and AUDIT-C showed a high predictive value.

The article "Nutrient intake, alcohol consumption, emotional eating and anxiety in women nursing students" was published in 2023. Journal: Heliyon.

Day consumption was measured with Standard Drink Units (SDU); in Spain SDU is 10 g. The alcohol consumption was divided into three categories: *Low-risk consumption* SDU ≤21 and ≤14 in men and women respectively), *Moderate-risk consumption* (22–27 and 15–16 SDU in men and women respectively) and *High-risk consumption* (≥28 and 17 SDU in men and women respectively). And binge-drinking in considered intake of ≥5 SDU per time [61].

c) Emotional Eater Questionnaire (EEQ)

This test consists of 10 items on a 4-category Likert scale from 0 (never) to 3 (always). The original validation with a sample of people with obesity [47] found three subscales: lack of control in eating, high calorie food preference, and feelings of guilt. Additionally, the test provides a global score of EE. The temporal stability shows medium-high correlation in the test-retest average (r = 0.702; p < 0.001) and the internal consistency of the subscales range from α = 0.61 to α = 0.77, what indicated the appropriate reliability of the instrument [62].

d) Anxiety

To measure levels of anxiety we used the State-Trait Anxiety Inventory (STAI) adapted by Guillen & Buela [63]. This questionnaire is composed of 40 items which evaluate two different concepts: anxiety as a state (a transitory emotional response) and anxiety as a trait (a constant anxious condition). The 20 items of each subsection use a Likert scale of categories from 0 (almost never) to 3 (very often/almost always). The analysis of psychometric properties of the instrument for university population showed a high internal consistency (α = 0.93) [35].

3. Statistical Analysis

Participants’ characteristics were examined using means, standard deviations (SD) and percentages. The matrix of correlations between variables was determined using the Pearson correlation coefficient between alcohol consumption, level of emotional eating and anxiety with nutrients and food intake.

## 3 Results

1 Descriptive Analysis of Nutrient intake, Emotional Eating and Food consumption

Differences were observed between students and with respect the intake of macronutrients. The energy intake of the diet in women nursing students reached only 78 % of the total energy intake in this sex and age group (Table 1). With respect the %E of alcohol, this percentage is good because they did not reach the maximum allowed. With respect protein intake we observed a high intake of them (211,5 %) intake upper the recommended intake of 41 g. The same result was obtained for %E of proteins, with 132.7 % of energy intake of proteins above the 15 % recommended. On the contrary, %E of carbohydrates is under the recommendations (55 %). Other energy sources were lipids with high intake of %E of total fat and %E saturated fatty acids (SFA), over the recommendations. Cholesterol intake is accordingly recommended values.

The article "Nutrient intake, alcohol consumption, emotional eating and anxiety in women nursing students" was published in 2023. Journal: Heliyon.

Micronutrient's intake appeared in Table 1; data was compared accordingly recommended Spanish dietary reference value (DRI). The nutrient intake under DRI were vitamins A, D, E, folic acid, Ca, Mg, K and Fe. And upper DRI of P and vitamins B_1_ and B_12_. Prevalence of adequacy for micronutrients intake (% population above 80 % RDI) in the study population is presented by age group and reporting in Table 1 according to Moreiras et al. [64].

Nursing women students were low emotional eater (44 %) > emotional eater (30 %) > non-emotional eater (22.7 %). In Table 2 were observed this population of students with respect their emotions. We observed that only 27 % were non emotional eater, the rest of students were affected by emotions.

**Table 1:** Daily intake of nutrients in nursing students.

Nutrient	Mean (SD)	*RDI* [65]	%RDI	P
*Energy (kcal)*	1792.8 (630.5)	2300	78.0	<0.01
*alcohol (g)*	10.4 (10.6)	<30	34.7	<0.01
*%E alcohol*	3.9 (3.9)	<10	39	<0.01
*P (g)*	88.3 (40.1)	41	215.4	<0.01
*g/kg P*	48.3 (9.1)	41	117.8	<0.01
*%E P*	19.9 (6.4)	15	132.7	<0.01
*CH (g)*	167.4 (73.1)			
*%E CH*	37.1 (8.3)	55	67.5	<0.01
*Fiber (g)*	20.9 (8.5)	25	83.6	<0.01
*Fat (g)*	73.6 (33.4)			
*%E Fat*	36.8 (9.5)	30	122.7	<0.01
*SFA (g)*	25.1 (11.8)			
*SFA%E*	12.5 (3.6)	<10	125	<0.01
*Cholesterol (mg)*	290.8 (127.1)	<300	96.9	0.05
*Vitamin D (μg)*	6.0 (3.9)	15	60	
*Vit. B*_*1*_*(mg)*	1.4 (0.6)	0.9	116.7	<0.01
*Vit. B*_*2*_*(mg)*	1.6 (0.6)	1.4	88.9	0.03
*B6 (mg)*	2.2 (0.8)	1.7	129.4	<0.01
*Folic acid (μg)*	257.0 (91.0)	400	64.3	<0.01
*Vit. B*_*12*_*(μg)*	4.8 (1.9)	2	240	<0.01
*Ca (mg)*	799.8 (272.0)	1000	79.9	<0.01
*Mg (mg)*	278.3 (79.5)	350	79.5	<0.01
*P (mg)*	1285.7 (437.0)	700	183.7	<0.01
*Fe (mg)*	12.9 (4.5)	18	71.7	<0.01
*K (mg)*	2701.5 (1078.8)	3500	77.2	<0.01

Data shows Mean (SD). RDI = recommended dietary intake. %RDI = disparity between reported consumption and the level needed for adequacy, calculated comparing with 80 % of the Spanish dietary reference value for macro and micronutrients.

**Table 2:** Classification of emotional eater in women Nursing students.

	Emotional eater
	%
*non-emotional eater*	22.7
*low-emotional eater*	42.0
*emotional eater*	30.4

In Table 3 we observed the intake of some different food-groups per day in nursing women students. In our students we observed that the intake of some foods were around 2–3 times per week: cereals, fruit, vegetables, eggs, meat, EVOO, fast food, juices, and soft drinks. On the contrary the intake of dairy products and legumes were once per week. With respect fast-food and meat derivative their intake is 2 times per week.

The article "Nutrient intake, alcohol consumption, emotional eating and anxiety in women nursing students" was published in 2023. Journal: Heliyon.

**Table 3:** Intakes per day of different foods in women students.

*Food intake:* mean (SD)	
*dairy and dairy products*	0.1 (0.1)
*eggs*	0.6 (0.4)
*meat*	0.3 (0.2)
*Meat derivative*	0.3 (0.2)
*fish*	0.3 (0.2)
*vegetables*	0.3 (0.2)
*fruits*	0.3 (0.2)
*nuts*	0.3 (0.3)
*cereals*	0.4 (0.3)
*legumes*	0.1 (0.1)
*EVOO*	0.6 (0.3)
*sweets*	0.2 (0.1)
*fast-food*	0.3 (0.2)
*soft drinks*	0.3 (0.3)
*juices*	0.3 (0.2)

In Table 4 we presented the results of Audit survey. The women students were mainly into low-risk consumption (82.7 %), with respect the second question of Audit: *How many drinks containing alcohol do you have on a typical day when you are drinking?* 90.7 % of the students drink between 1 and 4 drinks. And when they drink alcohol 59.1 % had more than 40 g alcohol.

2. Correspondence of Emotional Eating with respect Nutrient intake, Food consumption and Alcohol consumption

**Table 4:** Alcohol consumption in women students.

Alcohol consumption		N	%
AUDIT question 2	1 or 2	81	54
	3 or 4	55	36.7
	5 or 6	12	8
AUDIT	Alcohol education	124	82.7
	Simple advice	25	16.7
Alcohol intake (g)	nondrinkers	20	13.4
	0–20 g	16	10.7
	>20–40 g	25	16.8
	>40 g	88	59.1

In Table 5 women students showed and inverse correlation between emotional eating and the intake of calories (p < 0.05). We also detected an inverse correlation between emotional eating and the intake of proteins, carbohydrates and direct relation with AUDIT and alcohol consumption (p > 0.05).

**Table 5:** Bivariate correlations of Emotional Eater, Macronutrients and Alcohol in women students.

	calories	protein	HC	Fiber	FA	SFA	MUFA	PUFA	cholesterol	alcohol	AUDIT	EE
calories	–											
protein	,644**	–										
HC	,819**	,405**	–									
fiber	,402**	,505**	,382**	–								
FA	,689**	,325**	,541**	0,079	–							
SFA	,725**	,418**	,486**	0,118	,809**	–						
MUFA	,602**	,292**	,466**	0,094	,924**	,705**	–					
PUFA	,465**	,536**	,234**	0,127	,566**	,396**	,526**	–				
cholesterol	,341**	,340**	0,118	−0,021	,426**	,478**	,399**	,400**	–			
alcohol	0,065	0001	0,053	−0,045	0065	0,047	0,03	−0,091	−0,105	–		
AUDIT	0,066	0006	0,045	−0,061	0035	−0,013	0001	−0,036	−0,121	,813**	–	
EE	-,160*	−0,148	−0,111	−0,054	−0,014	−0,044	−0,039	−0,045	0099	0,093	0,14	–

*p < 0.05; **p < 0.01; EE: Emotional Eater; FA: fatty acids; SFA: saturated fatty acids; MUFA: monounsaturated fatty acids; PUFA: polyunsaturated fatty acids, HA: carbohydrates.

The article "Nutrient intake, alcohol consumption, emotional eating and anxiety in women nursing students" was published in 2023. Journal: Heliyon.

In Table 6 we observed in women students that emotional eating was inversely correlated with the intake of vitamin B1 and magnesium (p < 0.05). With respect AUDIT no significant correlation was detected, but inverse relation was obtained between vitamins B1, B2, B6, B9 and B12 with the alcohol consumption.

**Table 6:** Bivariate correlations of Emotional Eater, Micronutrients and Alcohol.

	AUDIT	EE	Vit. B1	Vit. B2	Vit. B6	Vit. B9	Vit. B12	Vit. D	Ca	Fe	Mg	Na	K	P
AUDIT	–													
EE	,140	–												
Vit. B1	-,023	-,178*	–											
Vit. B2	-,044	-,105	,522**	–										
Vit. B6	-,055	-,106	,696**	,581**	–									
Vit. B9	-,112	,012	,361**	,407**	,490**	–								
Vit. B12	-,031	-,027	,045	,122	,098	,089	–							
Vit. D	,042	,008	,031	-,129	-,075	-,179*	,162*	–						
Ca	,017	-,084	,358**	,528**	,331**	,370**	,129	-,095	–					
Fe	-,012	,041	,415**	,442**	,436**	,467**	,098	-,145	,355**	–				
Mg	-,029	-,185*	,325**	,298**	,330**	,365**	,073	-,046	,414**	,234**	–			
Na	-,036	,127	,043	,017	-,018	,154*	,163*	-,065	,117	,461**	-,023	–		
K	-,015	-,129	,516**	,203**	,513**	,492**	,109	-,068	,433**	,400**	,339**	,134	–	
P	,057	-,087	,481**	,487**	,479**	,322**	,194*	-,161*	,573**	,253**	,337**	,067	,429**	–

*p < 0.05; **p < 0.01; EE: Emotional Eater.

In Table 7 we studied the correlation between emotional eating and AUDIT accordingly the intake of some foods. It was observed that emotional eaters eat increased the intake of fast food and sweets. With respect to AUDIT, it was correlated with the intake of processed meat and fast-food. Also, it is having observed a strong correlation between students who take sweets with soft drinks, fast-food and juices (p < 0.001) and the emotional eating is significantly correlated with sweets and fast-food.

3 Correspondence of State and Trait Anxiety with respect Nutrients, Food Intake and Alcohol consumption

**Table 7:** Bivariate correlations of Emotional Eater, Food intake and Alcohol.

	AUDIT	EE	Meat	Processed meat	Fish	Vegetables	Fruits	AOVE	Sweets	Fast-food	Soft drinks	juices
AUDIT	–											
EE	,140	–										
Meat	,048	,019	–									
Processed meat	,182*	-,031	,286**	–								
Fish	,050	,125	,085	,074	–							
Vegetables	,024	-,035	,133	,019	,338**	–						
Fruits	,014	,172	,063	-,005	,244**	,183*	–					
AOVE	,035	-,050	,004	-,048	-,002	,165*	-,071	–				
Sweets	-,105	,173*	,099	,087	,128	,116	,163*	,093	–			
Fast-food	,158*	,212**	,034	,046	,176*	,103	,321**	-,083	,246**	–		
Soft drinks	,008	,023	,026	,067	,090	,059	,105	,022	,309**	,169*	–	
Juices	-,040	,049	,197*	,128	,055	,161*	,246**	-,046	,247**	,214**	,197**	–

*p < 0.05; **p < 0.01; EE: Emotional Eater. AOVE: extra virgin olive oil.

The article "Nutrient intake, alcohol consumption, emotional eating and anxiety in women nursing students" was published in 2023. Journal: Heliyon.

In Table 9 we analyzed alcohol consumption and anxiety with respect intake of macronutrients, fiber, and alcohol. With respect AUDIT it was correlated with alcohol intake. Anxiety was correlated with the intake of fat and mainly with MUFA.

**Table 8:** Bivariate correlations of Anxiety, Macronutrients and Alcohol.

	AUDIT	Anxiety trait	Anxiety state	Calories	Proteins	HC	Fiber	FA	SFA	MUFA	PUFA	Cholesterol	Alcohol
AUDIT	–												
Anxiety trait	,005	–											
Anxiety state	,001	,362**	–										
Calories	,066	-,067	-,061	–									
Protein	,006	,031	,017	,644**	–								
HC	,045	-,060	-,118	,819**	,405**	–							
Fiber	-,061	,143	-,035	,402**	,505**	,382**	–						
FA	,035	-,189*	-,058	,689**	,325**	,541**	,079	–					
SFA	-,013	-,136	-,023	,725**	,418**	,486**	,118	,809**	–				
MUFA	,001	-,157*	-,092	,602**	,292**	,466**	,094	,924**	,705**	–			
PUFA	-,036	-,110	-,026	,465**	,536**	,234**	,127	,566**	,396**	,526**	–		
Cholesterol	-,121	-,114	-,080	,341**	,340**	,118	-,021	,426**	,478**	,399**	,400**		
Alcohol	,813**	-,006	,015	,065	,001	,053	-,045	,065	,047	,030	-,091	-,105	

*p < 0.05; **p < 0.01; FA: fatty acids; SFA: saturated fatty acids; MUFA: monounsaturated fatty acids; PUFA: polyunsaturated fatty acids.

**Table 9:** Bivariate correlations of Anxiety, Micronutrients and Alcohol.

	AUDIT	Anxiety trait	Anxiety state	Vit. B1	Vit. B2	Vit. B6	Vit. B9	Vit. B12	Vit. D	Ca	Fe	Mg	Na	K	P
AUDIT	–														
Anxiety trait	,005	–													
Anxiety state	,001	,362**	–												
Vit. B1	-,023	,049	-,078	–											
Vit. B2	-,044	-,074	-,049	,522**	–										
Vit. B6	-,055	,053	-,062	,696**	,581**	–									
Vit. B9	-,112	-,011	-,084	,361**	,407**	,490**	–								
Vit. B12	-,031	-,034	-,001	,045	,122	,098	,089	–							
Vit. D	,042	,135	,066	,031	-,129	-,075	-,179*	,162*	–						
Ca	,017	-,082	-,047	,358**	,528**	,331**	,370**	,129	-,095	–					
Fe	-,012	-,144	-,128	,415**	,442**	,436**	,467**	,098	-,145	,355**	–				
Mg	-,029	,057	-,025	,325**	,298**	,330**	,365**	,073	-,046	,414**	,234**	–			
Na	-,036	-,090	-,002	,043	,017	-,018	,154*	,163*	-,065	,117	,461**	-,023	–		
K	-,015	-,050	-,041	,516**	,203**	,513**	,492**	,109	-,068	,433**	,400**	,339**	,134	–	
P	,057	,067	-,033	,481**	,487**	,479**	,322**	,194*	-,161*	,573**	,253**	,337**	,067	,429**	–

*p < 0.05; **p < 0.01.

In Table 8, we did not found correlations between alcohol consumption and anxiety with respect some micronutrients. Only we observed an inverse correlation between trait anxiety and fatty acids and MUFA intake.

The article "Nutrient intake, alcohol consumption, emotional eating and anxiety in women nursing students" was published in 2023. Journal: Heliyon.

In Table 9 no correlations observed between trait and state anxiety and AUDIT. In Table 10 in women nursing students a positive correlation was detected between AUDIT and intake of fast food and processed meat (p < 0.05). In Table 10 significant correlations was detected between respondents’ alcohol consumption and more intake of processed meat and fast food and between state anxiety and meat consumption.

**Table 10:** Bivariate correlations of Anxiety, Food intake and Alcohol.

	AUDIT	Anxiety trait	Anxiety state	Meat	Processed meat	Fish	Vegetables	Fruits	Sweets	Fast food	Soft drinks	Juices
AUDIT	–											
Anxiety state	,001	–										
Anxiety trait	,005	,362**	–									
meat	,048	,135	,198**	–								
Processed meat	,182*	,053	,109	,286**	–							
Fish	,050	-,014	,031	,085	,074	–						
Vegetables	,024	,101	,080	,133	,019	,338**	–					
Fruits	,014	,052	-,057	,063	-,005	,244**	,183*	–				
Sweets	-,105	,033	,069	,099	,087	,128	,116	,163*	–			
Fast food	,158*	,047	-,045	,034	,046	,176*	,103	,321**	,246**	–		
Soft drinks	,008	,029	,009	,026	,067	,090	,059	,105	,309**	,169*	–	
Juices	-,040	,133	,100	,197*	,128	,055	,161*	,246**	,247**	,214**	,197**	–

*p < 0.05; **p < 0.01.

## 4 Discussion

The aims of the study were to analyze dietary habits, alcohol habits, emotional eating, and anxiety in a women Spanish university sample and to determinate if anxiety and emotional eating were related to dietary habits.

In our study, diet was evaluated throughout a three-day record and was observed differences according to their intake of nutrients, which respect the caloric intake for macronutrients was unbalanced (higher for proteins and lipids and lower for carbohydrates) and under the DRI: vitamins A, D, E, folic acid and Ca, Mg, K, Fe. Similar results were observed in other studies in university students, in which the typical diet described for Spanish population tends to be rich in protein/fat, specially saturated fat, cholesterol and poor in carbohydrate and fiber [[66], [67], [68], [69], [70], [71], [72], [73]]. According to a qualitative survey conducted by German university students, they frequently overestimate their knowledge on nutrition when using a quantitative questionnaire and they found that the students after an exhausting university day, were no motivated to spend time on cooking a healthy meal. Additionally, they discovered that students did not fully understand what a good diet entailed and that they needed more information on this topic [2]. Nursing students need to have a solid understanding of nutrition and its impact on health. By having healthy nutrition habits, they can better apply that knowledge in their clinical practice. Furthermore, by personally experiencing the benefits of proper nutrition, they can effectively convey that knowledge to their patients.

The article "Nutrient intake, alcohol consumption, emotional eating and anxiety in women nursing students" was published in 2023. Journal: Heliyon.

In the current study, we found that various foods were consumed around 2–3 times per week: cereals, fruit, vegetables, eggs, meat, fast food, juices, and soft drinks. Similar findings were found among Spanish university students, 79 % of whom did not meet the daily recommendation of 5 servings of fruits and vegetables for health [3,65]. With respect the intake of dairy products and legumes were once per week and fast-food and meat derivative intakes were 2 times per week. Our results differ with ANIBES in Spanish population [5].

Emotional eating may require that people learn to associate emotion with eating, may follow only specific discrete emotions and may depend on social context [57]. The present study showed that nursing women students were low emotional eater (44 %) > emotional eater (30 %) > non-emotional eater (22.7 %). We reported similar findings in a prior study conducted among students of health sciences, in which 40.4 % were low emotional eaters, 29 % were emotional eaters and 28.2 % non-emotional eaters [74]. Emotional eating in our students is significantly correlated with sweets and fast-food, that is, with less healthy food intake patterns. As in our results, previous studies show that emotional eating is associated with higher intakes of snack/fast-food and higher total energy intake [75].

Participants of our study showed a correlation between AUDIT and intake of fast food and processed meat (p < 0.05), and we did not find a reduction in caloric intake with drinking. Similar findings were observed in a qualitative study that explored the links between alcohol intake and unhealthy eating behavior, evidencing that young adults consume high-calorie food products when drinking [76].

The prevalence of alcohol intake among female university students in different countries were 28.1 % in Bulgaria, 18.1 % in Germany, 10 % in Poland [9]. In Japan approximately 47.8 % of female university students were binge drinkers and alcohol was the most abused substance by university students in the United Kingdom and Ireland [11,77]. In the present study 82.7 % of women students were into low-risk consumption, according to AUDIT test. Similar findings were found in a prior study by Marchena et al. (2020) in Spanish health sciences university students, in which 80 % of participants can be considered as not at risk of alcohol consumption [55,78]. 59.1 % of the students normally took1-4 alcoholic drinks, and into this group one of the participants had more than 40 g alcohol (59.1 %). It has been suggested that drinking behavior depends on the time spent in the university, t [79]he longer the period a student spends in the university, the higher his/her risk of drinking [80].

The article "Nutrient intake, alcohol consumption, emotional eating and anxiety in women nursing students" was published in 2023. Journal: Heliyon.

Some authors reported that anxiety rate is increasing rapidly [81] among university students [82] and that anxiety contributed to develop disordered eating [83], disorders that are more prevalent in female population [84]. In line with several recent investigations amongst university students it has been observed a desire for thinness among male and female university students [[84], [85], [86]]. In a cross-cultural study involving female students, 8.6 % of the Russian and 7.9 % of the Japanese respondents appeared at risk and 6.8 % of Hong Kong and Chinese adolescents girls have eating disorders 2022 [81,87]. Eating problems in university students are associated with a range of deleterious consequences including lower academic functioning [87]. Eating disorders observed in undergraduate students in different countries: 8.9 % in Poland [88], 11.3 % in Croatia [89], 12.64 % in the United States [83] and 20.8 % in Spain [90]. In our study EE, was correlated with the intake of calories and fast food, on the contrary state and trait anxiety was not correlated with nutrients or the intake of some foods. López Olivares et al. (2020) observed that anxiety was linked with the more caloric foods as coping strategy [13]) as the intake of unhealthy food can become an important reinforcer [14]. In a previous study developed in students of Health Sciences, Marchena et al. (2020) explained that state-anxiety is more associated with specific external situations and is more susceptible to change than trait anxiety, by changing stressful contextual factors or implementing appropriate coping strategies. It is important to take these differences into account when designing prevention/intervention strategies and profiles of unhealthy eating habits [55].

In the present study the diet was evaluated throughout a three-day dietary, similarly to that the ANIBES study used the same proceeding [15]. Differences were observed between students and with respect the intake of macronutrients. The energy intake of the diet in women nursing students reached only 78 % of the total energy intake in this sex and age group (Table 1). With respect the %E of alcohol, this percentage is good because they did not reach the maximum allowed. With respect protein intake we observed a high intake of them (211,5 %) intake upper the recommended intake of 41 g. The %E of proteins, was 132.7 % above of recommendations. On the contrary, %E of carbohydrates is under the recommendations (55 %). Other energy sources were lipids with high intake of %E of total fat and %E saturated fatty acids (SFA), over the recommendations. Cholesterol intake is accordingly recommended values. Micronutrient's intake appeared in Table 1 data was compared accordingly recommended Spanish dietary reference value (DRI). The nutrient intake under DRI were vitamins A, D, E, folic acid, Ca, Mg, K and Fe. And upper DRI of P and vitamins B1 and B12. In the Spanish ANIBES population it has been also observed elevated intakes of SFA and under nutrient requirements for fiber, Ca, Zn, folic acid and vitamins A and C [91].

The article "Nutrient intake, alcohol consumption, emotional eating and anxiety in women nursing students" was published in 2023. Journal: Heliyon.

Nursing students should practice healthy lifestyle habits not just to offer their patients with high-quality care, but also because they are expected to set an example for their patients and the community at large as future healthcare professionals. Additionally, preserving strong physical and mental health lowers the chance of burnout, which is essential for a long-lasting and satisfying nursing job.

This study has several limitations. First, it was a cross sectional study. Second, we could not obtain sociological data such as the family's socioeconomic status or the parents' academic history. Another limitation was the total sample of the students, because over 20 % of the recruited participants finally did not agree to be included in the study.

## 5 Conclusions

The healthy nursing women students' eating index (HEI) was insufficient. The calorie intake for the macronutrients were below the DRI and imbalanced (greater for proteins and lipids and lower for carbohydrates) and under the recommendations for micronutrients: vitamins A, D, E, folic acid and Ca, Mg, K, Fe.

This study suggest that nursing students tended to be low emotional eaters (44 %) compared to emotional eaters (30 %) and non-emotional eaters (22.7 %). Significant links exist between EE and eating fast food, sweets, or engaging in other unhealthy eating habits.

Finally, 82.7 % of female students reported low-risk regular alcohol intake, however the more drinker students the unhealthier eating behavior had. 79 % did not reach the recommended intake of 5 serving/day of fruits and vegetables and greater intake of fast food and processed meat.

That's why future interventions should be necessary in university students, to future health promotion interventions and behaviors change in that young adult's population.

This study has some limitations. First, it was a cross-sectional study. Second, we could not obtain sociological data such as the family's socioeconomic status or the parents' academic history. Another limitation was the total sample of the students, because over 20 % of the recruited participants finally did not agree to be included in the study.

The article "Nutrient intake, alcohol consumption, emotional eating and anxiety in women nursing students" was published in 2023. Journal: Heliyon.

## Funding

This research was supported by 10.13039/100012986Universidad Francisco de Vitoria (10.13039/100012986UFV 2022–26).

## Data availability statement

No data associated with your study been deposited into a publicly available repository.Data will be made available on request.

## CRediT authorship contribution statement

**María Teresa Iglesias López:** Writing – review & editing, Writing – original draft, Validation, Investigation, Formal analysis, Data curation, Conceptualization. **Carlos-Alberto Marchena-Giráldez:** Writing – review & editing, Writing – original draft, Validation, Supervision, Software, Methodology, Investigation, Formal analysis, Data curation, Conceptualization. **Elena Bernabéu-Brotons:** Writing – review & editing, Writing – original draft, Validation, Supervision, Resources, Project administration, Methodology, Investigation, Funding acquisition, Formal analysis, Conceptualization.

## Declaration of competing interest

The authors declare the following financial interests/personal relationships which may be considered as potential competing interests.
